# MRI Radiogenomics in Precision Oncology: New Diagnosis and Treatment Method

**DOI:** 10.1155/2022/2703350

**Published:** 2022-07-07

**Authors:** Xiao-Xia Yin, Mingyong Gao, Wei Wang, Yanchun Zhang

**Affiliations:** ^1^Cyberspace Institute of Advanced Technology, Guangzhou University, Guangzhou 510006, China; ^2^Department of Radiology, The First People's Hospital of Foshan, Foshan 528000, China; ^3^Pengcheng Laboratory, Shenzhen, China

## Abstract

Precision medicine for cancer affords a new way for the most accurate and effective treatment to each individual cancer. Given the high time-evolving intertumor and intratumor heterogeneity features of personal medicine, there are still several obstacles hindering its diagnosis and treatment in clinical practice regardless of extensive exploration on it over the past years. This paper is to investigate radiogenomics methods in the literature for precision medicine for cancer focusing on the heterogeneity analysis of tumors. Based on integrative analysis of multimodal (parametric) imaging and molecular data in bulk tumors, a comprehensive analysis and discussion involving the characterization of tumor heterogeneity in imaging and molecular expression are conducted. These investigations are intended to (i) fully excavate the multidimensional spatial, temporal, and semantic related information regarding high-dimensional breast magnetic resonance imaging data, with integration of the highly specific structured data of genomics and combination of the diagnosis and cognitive process of doctors, and (ii) establish a radiogenomics data representation model based on multidimensional consistency analysis with multilevel spatial-temporal correlations.

## 1. Introduction

Tumor heterogeneity, one of the main characteristics of malignant tumors, poses great challenges to its accurate diagnosis and treatment, which is also manifested by multiple genotypes and multiple gene expression patterns in the same tumor cells [1]. The same tumor presents distinctly different therapeutic effects and prognosis in different individuals, and even tumor cells in the same individual present varied characteristics though with the same genome [2]. As shown in Figure 1, tumor heterogeneity is manifested in both space and time. In terms of space, the combined effects of molecular variation and tumor microenvironment lead to differences in tumor regions [3], which can be classified as follows: (i) intertumor heterogeneity, that is, differences between tumors in different patients; (ii) intratumor heterogeneity, that is, completely different or even opposite patterns of the expression patterns of cells in different tumor regions, which may result in the changes in structure and differential responses to therapeutic drugs [4]. In terms of time, tumor is a dynamic system, and tumor cells evolve over time with multiple variations and temporal heterogeneity, which requires the reproducible detection in time. However, current genomics technology is static and can only reflect the information of a point (snapshot) on the time axis. Current molecular profiling analysis on locally extracted tumor tissue**s** at a single time point reflects only a small part of the information of the entire tumor in both the spatial and temporal dimensions and fails to fully analyze the characteristics of the tumor. Quantitative description of tumor heterogeneity may lead to one-sided or even erroneous diagnosis, affecting the treatment options, and leading to drug resistance and disease recurrence in patients.

Genome analysis technology attempts to solve the problem of tissue sampling and analysis under tumor heterogeneity, such as the multiregion sampling strategy for spatial heterogeneity, and the micro-cutting of different tumor tissues for the isolation of small tissue fragments. DNA of these fragments has been analyzed [6]. However, this method requires precise localization of the tumor area during sampling to ensure the sampling genes obtained coming from tumor cells, which greatly limits the success rate of such a method. Longitudinal sampling attempts to solve the problem of temporal heterogeneity. Pathological sections are obtained at different stages of tumor treatment to track the variation of tumor-related genes and accurately analyze tumor heterogeneity [7–9]. However, the longitudinal sampling method requires multiple acquisition of patient tissue samples, and the invasive nature of this method terribly limits its feasibility in clinical practice. In short, the heterogeneity of tumors brings considerable challenges to precise diagnosis and treatment. Merely relying on linear, invasive, and single-time-point genomics technology cannot well meet the needs of precise clinical diagnosis and treatment, making it necessary to explore a three-dimensional, noninvasive, and reproducible method.

Broadly speaking, tumors are made of evolved and heterogeneous populations of cells that are resistant to matched targeting therapy. Thus, it is not enough reliable to evaluate effects of tumor treatment and diagnosis only from the perspective of tumor abnormality [10, 11]. Tumor genome analysis has been the gold-standard technique for molecular mapping [12, 13]. Nevertheless, the study on genomic heterogeneity has revealed that individual tumor may be clonally independent without shared driver gene alterations [14]. There is a proof-of-concept study demonstrating that morphological heterogeneity reflects structural and functional divergence. Moreover, there is a close link between morphological phenotypes and stromal and cancer-cell-related features that allow prediction of the morphological pattern [15]. Furthermore, a better understanding of the molecular background is conducive to preventing adverse drug reactions for defined patient groups [16, 17]. However, drug therapy matched to the molecular target does not necessarily produce positive results [18, 19]. This is affected by multiple factors such as tumor microenvironment and tumor heterogeneity. In summary, the foregoing findings demonstrate that the genetically, morphologically, phenotypically, and topologically distinct primary cancers can not only be present in an individual patient but also are of great significance to personalized medicine approaches, as they can limit therapeutic efficacy, and they are resistant to therapy.

This paper was aimed at reviewing the methods in literature regarding the precise diagnosis and prognosis prediction of neoadjuvant chemotherapy for tumors, using breast MRIs, for example. Taking tumor heterogeneity as the core issue, the deep learning-based radiogenomics analysis of breast tumor heterogeneity was studied, and the relationship between the imaging characteristics of heterogeneous tumors and molecular expression features was correspondingly explored as well. At the same time, geometric algebra was applied to design a framework for analyzing dynamic contrast enhanced MRI radiogenomics, and fully mining the rich spatial images, spatial signals, and semantic features in breast multidimensional magnetic resonance imaging. According to the heterogeneity of different tumors, an individualized model of neoadjuvant chemotherapy efficacy prediction was established by combining MRI information, molecular typing information, and clinical information of patients suffering from breast cancer, which provided scientific guidance for accurate diagnosis, treatment, and prognosis of patients, improved the survival rate of tumor patients, enhanced the life quality of patients after surgery, and achieved effective and rational utilization of medical resources.

The remainder of the paper is structured as follows: Section 2 discusses challenges in the analysis of tumor heterogeneity using radiogenomic approaches; the main framework for radiogenomics analysis in literature is presented in Section 3, where the mathematical models applied for tumor diagnosis and the evaluation of tumor treatment and prognosis performance via multiomics are presented; Section 4 addresses outlook and future work, where a multilevel deep learning model named BiGRU-RNN is proposed for predicting the efficacy of neoadjuvant chemotherapy using radiogenomics. It is represented by introducing geometric algebra and enables the multidimensional unified analysis of dynamic contrast enhanced MRI radiogenomics; finally, Section 5 summarizes the most significant parts in each section in a simplified manner.

## 2. Challenges in the Analysis of Tumor Heterogeneity Using Radiogenomic Approaches

In biomedical analysis, tumor heterogeneity characteristics and multiple physiological tumor characteristics are not combined, and multimodal (parametric) imaging technology is not widely used [20]. Various “spectrum” analyses of images from different perspectives describing these physiological characteristics have led to the one-sidedness and singularity of the research. In addition, current radiogenomics analysis on tumor heterogeneity assumes that the voxel of each tumor image presents a single specific tissue characteristic. However, tumors are highly heterogeneous. Current resolution of clinical diagnostic images is rather finite, and the observed signal at a certain position (voxel) of the tumor may be a mixture and superposition of components of different characteristics [21, 22]. From the perspective of signal processing, tumor image heterogeneity is manifested as a multivariate (component) mixed signal processing problem. In this regard, a lot of preliminary researchers work on the DCE-MRI subcomponent decomposition [23, 24], the corresponding molecular information decomposition [25, 26], and an unsupervised convex analysis analyzing the components of different tissue characteristics of heterogeneous tumors [6]. These researches afford a further understanding of the physiology and molecular characteristics of tumors.

At present, this method is only applied for two-dimensional analysis of DCE-MRIs [27–29], and there is no further development of heterogeneous analysis of tumors based on three-dimensional multi-modal MRIs [30–32]. The radiogenomics issues such as the correlation between different subcomponents after decomposition and the application of tumor diagnosis and treatment also need further exploration. Additionally, current heterogeneity analysis and subregion/subcomponent decomposition research mainly focus on the tumor itself, ignoring the fact that tumor does not exist in isolation, which constantly exchanges information with the surrounding substance and microenvironment during the growing process, and is also affected by the surrounding substance. Tumor cells can reshape the microenvironment, and the changed microenvironment can further affect the behavior and status of tumor cells, leading to tumor progression and metastasis. Therefore, the formation of tumor heterogeneity is the result of the joint action of the tumor body and its surrounding substance. Currently, heterogeneity analysis is mostly limited to the structure and function of the tumor itself, and there is few literatures reporting the heterogeneity of tumor stroma [33, 34].

In recent years, there have been several researches concerning the radiomics research of tumor stroma. For example, King et al. found that the increase in the dynamic enhancement rate of fibroglandular mammary glands was associated with higher mammary cancer morbidity [35], who divided the body into several band-shaped regions according to the distance from the tumor and investigated the relationship between these regions and the disease-free survival of breast cancer [36]. However, the analysis of tumor heterogeneity in these studies was still preliminary, qualitative, or semiquantitative analysis. No systematic work has been performed to quantitatively analyze the relationship between the tumor and the surrounding substance or analyze the heterogeneity of the substance. In addition, the analysis of tumor heterogeneity in radiogenomics research at this stage generally focuses on image feature analysis. The collected gene molecular information is assumed to be homogeneous by default, but in fact, the tissue collected in molecular expression analysis may be a mixture of tissues with different “content” and different characteristics [37]. Besides, current radiogenomics research does not analyze the heterogeneity of the tumor itself, resulting in the inaccuracy of the associated study, and even the appearance of “false relationships.” Previous research was conducted in terms of signal subcomponent decomposition analysis, biological verification research on gene expression values of different tissue characteristics (human brain, liver, and lung), and unsupervised identification of mixed tissue characteristics [31, 32]. The gene expression signal of heterogeneous tumors has not been further analyzed. Therefore, the research of radiogenomics based on the decomposition of gene information is urgently required.

## 3. Methodology of Radiogenomics in Literature

As a noninvasive modality, the multidimensional radiogenomics analysis based on Magnetic Resonance Imaging (MRI) has become a special field of study on the tumor grading. The field of radiogenomics has been advanced substantially by novel MR imaging sequences that reflect underlying oncogenic processes. MRI-based radiogenomics combines a mass of quantitative data extracted from multidimensional MR images with individual genomic phenotypes and builds a prediction model through deep learning, which aims to make a diagnosis for patients, offer guidance for therapeutic strategies, and make an evaluation on clinical outcomes [38]. Additionally, some issues existing in radiogenomic analysis are specified, and corresponding solutions from prior works are provided [39]. Illustratively, the abundance of immune and stromal cells in the Tumor Microenvironment (TME) indicates the levels of inflammation, angiogenesis, and desmoplasia. It has been proven that radiomics, an approach of extracting quantitative features from radiological imaging to characterize diseases, can predict molecular classification, cancer recurrence risk, etc. However, the ability of radiomics to predict the abundance of various cells in the TME remains unknown. Arefan et al. [40] carried out studies by applying a radiogenomics approach and building machine learning models to capture one-to-one relationships between radiomic features from Dynamic-Contrast Enhanced Magnetic Resonance Imaging (DCE-MRI) and cell abundance of gene expression data and then predict the infiltration of multiple cells in breast cancer lesions. It is concluded that radiogenomics contributes to computer-aided diagnosis, treatment, and prognostic prediction for patients with tumors in a routine clinical setting.

### 3.1. Tumor Diagnosis Research Based on Radiogenomics

Radiogenomics, as an important application, reveals and reflects the molecular pathological characteristics of tumor tissues, such as dynamic enhancement characteristics for tumor and mammary-gland tissue [33, 34] and breast asymmetry characteristics [34] in distinguishing benign and malignant tumors using noninvasive and dynamic imaging technology.

Tumor molecular classification is an important index in clinical diagnosis. In several studies, quantitative image features, such as the dynamic enhancement ratio of the lesion to the background area, gray-scale histogram features, and 66texture, are used to predict these molecular indicators [37, 41]. It has been reported that there are 90 extracted image features, including the morphology, dynamic enhancement, and bilateral asymmetry of breast cancer tumors and their background regions, all of which are used to distinguish four molecular subtypes of breast cancer [42]. In recent years, radiomics features, including tumor volume, shape, edge morphology, and dynamic characteristics, have also been used to predict the expression of gene chips for clinical diagnosis, such as MammaPrint, Oncotype DX, and PAM50 gene arrays [43–45]. Additionally, some researchers have studied the MR image characteristics of breast cancer in the TCIA database and the molecular information such as miRNA, gene somatic mutation, protein expression, and copy number variation of these patients in the corresponding TCGA database. It has been found that there are several genetic signaling pathways, gene mutation sites, and image feature modules significantly related to gene expression modules [46]. The above-mentioned study in image group characteristics and gene expression correlation is to explore the imaging biomarkers of tumor molecular characteristics, thus providing services for clinical diagnosis [47].

### 3.2. Tumor Treatment and Prognosis Research Based on Imaging Group Feature Analysis

Currently, a large amount of research regarding radiogenomics focuses on exploring the relationship between imaging group and molecular features. Some work bypasses the association between imaging and molecular information and directly uses imaging features to predict treatment results.

It has been investigated that the imaging phenotype of the tumor can be used to provide information on the outcome of tumor treatment, such as chemotherapy efficacy and prognosis. Fan et al. extracted 156 image features of breast tumors and background regions using DCE-MRIs and selected several distinguishing heterogeneous features reflecting gray-scale unevenness, such as kurtosis and skewness, to predict the effectiveness of NAC for breast cancer [48]. Huang et al. extracted the gray-scale texture features of colorectal cancer images to predict lymph node metastasis (disease-free survival) before surgery [49]. Some researchers used cluster analysis to divide the imaged tumor into different regions according to the dynamic enhancement mode, analyzed the differences in the texture characteristics of these regions before and after chemotherapy, and predicted the efficacy of chemotherapy using the detected features [26], proving that the imaging characteristics of different tumor areas could be used to predict the efficacy of NAC. Additionally, key tumor genes were detected and identified by analyzing the differences in the network structure of the tumor genome before and after treatment, combined with the analysis of the tumor volume growth pattern of MRIs in terms of its longitudinal time, to predict the treatment response of tumors [50].

With the use of perfusion magnetic resonance (MR) imaging, Wu et al. characterized intratumoral spatial heterogeneity and studied the tumor homogeneity to predicate the recurrence-free survival (RFS) of the patients with breast cancer [51].  Figure 2 proposed a two-stage intratumor partition framework, including stage I: individual level cluster; and stage II: population level cluster. Primarily, at a personal level, every tumor is exceedingly segmented via superpixels using four kinetic features, that is, percentage and signal enhancement ratios, as well as the wash-in and wash-out slopes, according to DCE-MRIs [52–54]; secondly, at the population level, a consensus cluster can be used to aggregate and uniformly mark all superpixels from the entire population. Additionally, it is possible to establish the congruent relationship between tumor subregions across patients among the given population. Breast cancer is constituted by several subregions with different spatial features, and the intratumoral spatial heterogeneity is characterized and quantified via the defined multi-regional spatial interaction (MSI) matrix. As a distinct independent prognostic factor, imaging heterogeneity is beyond those traditional predictive risk factors; similar radiogenomics is also used for predicting NAC efficacy [50, 55–57], prognosis [26, 48], survival period [58], distant metastasis [59], etc. However, most tumor treatments based on radiogenomics regimen only focus on describing and analyzing the overall gray-scale unevenness (texture, etc.) of imaged tumors [43], and the influence for diagnosis and treatment is rarely analyzed and measured in terms of the subregions (components) of heterogeneous tumors [44].

### 3.3. Tumor Treatment and Prognosis Research Based on Multiomics Approaches

Apart from the mentioned analysis of imaging group features, some researchers have also attempted to establish a multiomics approach for tumor diagnosis and treatment by combining image features and molecular features. For example, it was found that imaging methods exhibited different prediction results for patients with different molecular subtypes of breast cancer. Specifically, HER2-positive breast cancer was found to have a higher accuracy rate for its NAC treatment, while human epidermal growth factor receptor 2 (HER2) and triple-negative breast cancer (TNBC) had a lower accuracy rate [60], since patients with HER2-NBC and TNBC types presented high heterogeneity. During the establishment of tumor diagnosis and treatment models, intrinsic molecular characteristics shall be combined (HER2, etc.) to increase prediction accuracy. Sutton et al. found in the study of predicting breast cancer molecular subtypes based on image features that the accuracy of the model was significantly improved after adding clinical data and pathological data, including age of patients, tumor volume, tumor pathological grade, and accumulation of lymph node [61].

It was revealed that imaged tumor features and patient symptoms could be complementary, and the combination of the two could improve the accuracy of the prediction model. Although researchers have made considerable efforts on tumor diagnosis and treatment based on the analysis of clinical and molecular pathology information and image characteristics, there are few results in the research of precision diagnosis and treatment models combining the two features, and the methods and technologies in this area shall be studied and resolved. Besides, repeatability and reproducibility are the two relatively major problems [62] regarding radiogenomics analysis. The former refers to the consistency of multiple measurements under the same environment and experimental conditions, while the latter denotes that of grouped image features in different locations, imaging parameters, and experimental subjects. Solutions to these two problems, especially the latter, are the key to the radiogenomics diagnosis and treatment model, which requires the combination of theory and practice. Although some scholars have made exploratory attempts in this regard, such as the use of validation sets to analyze the consistency of radiogenomics [63], there are still few basic methods of radiogenomics, especially tumor heterogeneity analysis, radiogenomics study, and evaluation of the application of scientific methods and models in clinical tumor diagnosis and treatment.

Tumor heterogeneity poses challenges to the precise diagnosis and treatment of breast tumors. Its systematic analysis provides extensive information for the characterization of breast tumors, and effective application of this information is of great significance to improve the accuracy of breast cancer diagnosis and treatment. Fan et al. [48] explored the heterogeneity of tumors by analyzing the subclones with a mass of gene modifications and functional effects, which offered a deeper understanding of the method to identify the bioactivity of certain subclones with a radiogenomic analysis, and predicted the prognosis noninvasively and clinically.

Besides, a modelling framework was proposed by Fan et al. [48], as shown in Figure 3, where multiscale intratumor heterogeneity was modelled, and the radiogenomic analysis was carried out regarding 1310 patients suffering from breast cancer on 5 datasets of 3 data groups. This modelling framework consisted of three phases. Firstly (Phase 1), a nonsupervision deconvolution analysis on gene expression profiles was adopted to achieve genomic subclones, including prognostic genomic signatures; secondly (Phase 2), radiogenomic genomic characterization was established by means of mapping radiomic features onto compositions of prognostic subclones in an independent dataset containing the suited imaging and gene expression data from each tumor; thirdly (Phase 3), the predicated value of the recognized radiogenomic signatures was further investigated using another two independent datasets containing imaging and survival data. The findings provided a noninvasive and reproducible method to be used to identify tumor genomic subclones and their underlying biological clinical functions.

Table 1 is designed to intuitively classify and introduce the mentioned radiogenomics techniques and approaches in literature for diagnosis, treatment, and prognosis research.

## 4. Outlook and Future Work

Based on the radiogenomics techniques, this section aims to develop novel multidimensional mining algorithms, focusing on the key core issue of tumor heterogeneity. The proposed algorithms will lead to the identification of tumor patterns in complex geometric spaces. Through the analysis of multimodal images and molecular information reflecting different functional characteristics of tumors, we aim (1) to deeply mine the spatial, temporal, and semantic features of breast multidimensional images across scales; (2) to reveal the relationship between the overall and regional imaging phenotypes of tumors and recognize their joint functional characteristics with gene expression together with molecular typing; (3) to provide new intelligent solutions for breast tumor clinical diagnosis and neoadjuvant chemotherapy efficacy prediction, which can effectively assist doctors to make correct treatment decisions and improve patients' health.

### 4.1. Temporal-Spatial Consistent Correlation Model Based on MRI Radiogenomics

According to different description methods for tumor heterogeneity, the analysis on tumor radiogenomic correlation is to be carried out at three levels, that is, analysis of the whole tumor region, tumor subregions, and tumor subcomponents; regarding a single time point; and longitudinal time axis. Different levels of tumor heterogeneity can be mapped using geometry algebraic decomposition in relation to the multidimensional image space, image subspaces in different directions corresponding to the same dimensional image vector, and the cross-dimensional image signal vector features in different directions.

It is a crucial basis for accurate analysis of radiogenomics to realize the rapid and automatic parameter extraction of unstructured breast radiomics data and the effective fusion of unstructured feature vectors with diagnostic value found in structured data.

Based on the theory of geometric algebra, tumor images with different structures are transformed from complex geometric objects to straightforward geometries like dots, lines, and polygons that can be directly expressed in Euclidean space, so as to realize the hierarchical decomposition of the complex geometric data of breast tumors. Appropriate image segmentation and deep clustering methods should be adopted to analyze multiple geometric vectors in different dimensions. The final aim is to achieve deep learning and feature extraction of tumor heterogeneity based on multidimensional uniformity analysis in a multivector space and achieve the transition from unstructured imaging to structured genomics data.

As discussed in [64], it is easy to extend a scalar product to Clifford or geometric product to explain errors caused by patient movement, extract nonlinear features from images, or clarify observed scaling changes across the dimensions of a tumor, as illustrated in Figure 4.

### 4.2. Deep Association Learning between MRI Radiomics and Genomics

There are three parts proposed below for further realization of the deep association learning between MRI radiomics and genomics, as illustrated in Figure 5.

#### 4.2.1. Global Heterogeneity Analysis via the Correlation between Image and Molecular Features

Weak supervision can facilitate the acquisition of the datasets marked manually. Weak supervision learning enables the application of inexpensive weak labels, and such labels can be exploited to build a powerful prediction model. The overall heterogeneity of tumors can be measured, analyzed, and classified using weakly supervised learning [66–69] of imaged tumors. Weakly supervised spatial clustering can be used to sort the decomposed subregions according to the value of the cluster center position.

Taking DCE-MRI as an example, the clustering results of the initial enhancement speed and the later decline speed of the enhancement curve can be sorted out to obtain several (*i*) “omics” features, and this process for all tumor images (*j*) can be sorted out to obtain an *i* × *j* matrix, so that feature calculation and classification research can be performed on the same time signal dimension.

Meanwhile, in view of the characteristics of biomedical functions reflected in tumor images, it is proposed to study the correlation based on multimodal (parametric) image features and molecular analysis features. In order to comprehensively analyze the heterogeneity of different functional characteristics of tumors, image registration [70–73] is performed for calculating different functional images of tumors, including DCE-MRI and DWI, to obtain multiple “dimensions,” which means that each pixel point corresponds to dynamic characteristics, diffusion characteristics, etc. Such characteristic can be further used to calculate high-dimensional characteristics of imaged tumor heterogeneity and their correlation with molecular fractal characteristics.

#### 4.2.2. Correlation between Heterogeneous Image and Molecular Features via Subdomain Decomposition

To fully analyze the correlation between heterogeneous image features and molecular features, the mixed images and gene molecular expression signals are suggested to be decomposed separately. This practice is to realize high- and multidimensional vector analysis in an integral space, also the multidimensional subspace region analysis, and spatial-temporal consistency analysis of heterogeneous subcomponents. The goal is to establish correlation models at different levels and achieve more accurate relationship to highlight key entities for the image or signal processes and the relationship between multiple entities (spatial-temporal) in multidimensional vector space or subspace.

Simultaneously, the gene expression data can be analyzed using subpathways, submodules, and enrichment methods, thereby dividing them into several representative pathways, marked modules, and gene clusters. The expression signal is expected to break down according to different tissue and cell characteristics using the signal decomposition method, which will in turn constitute a “convex hull,” each containing some “marked” genes [74].

In order to study the correlation between characteristic components in terms of different tissues, the correlation between the subregions (components) of the tumor heterogeneity should be analyzed and sorted by the spatial-temporal consistency-based algorithm after the decomposition of the image group and gene expression data, as shown in Figure 5. Taking the dynamic enhanced image as an example, it is supposed that there are three subcomponents with different tissue features sorted into three levels according to the enhancement curve of each subcomponent after decomposition, that is, fast blood flow, medium blood flow, and slow flow velocity.

Each sample is decomposed into these three types of subcomponents, and then the radiogenomic association of each subcomponent (fast, medium, and slow) is analyzed separately for all samples. Unlike traditional analysis methods, the attention-based deep learning network aims to study and analyze the correspondence between high-dimensional image vectors and gene expression subcomponents and try to obtain more accurate map of relationships based on the relationship between “pure” subcomponents with the directions of themselves.

#### 4.2.3. Bidirectional Threshold Recurrent Neural Network (BiGRU-RNN) Model

The effective embedding of radiomics and genomics information plays a key role in establishing spatial-temporal consistent model of radiogenomics. The genomics information of breast multi-dimensional dynamic imaging is intricate, including image sequence information, and time series information, both unstructured data of magnetic resonance imaging and structured vector of genomics. The design of gated loop unit with memory mechanism is important not only for timing information, but also for the memory and integration of image and genomics information.

Therefore, the two-way activation embedding method of the gated cyclic unit is designed based on the lightweight Bi-GRU, and the activation gate is introduced to process the genomics data of breast cancer patients with individual differences. The AuGRU model enables effective fusion of the genome sequence-related output and tumor heterogeneity analysis via radiogenomics, along with molecular typing for classification.

Additionally, it is of importance to design a bidirectional threshold recurrent neural network (BiGRU-RNN) model based on memory and attention mechanism, which highlights tissue-level radiomics feature input and molecular typing feature vector and encodes the contextual interaction mechanism of the genomics feature vector of tumor. Such a model plays a key role in carrying out the effective correlation of the spatiotemporal features of dynamic images and constructing a joint representation model of image data and genomics data. The schematic diagram summarizing the proposed attention-based BiGRU-RNN network model is shown in Figure 6.

## 5. Discussion

Radiogenomics characteristics reveal multiscale intratumoral heterogeneity concerning biological functions and survival in breast cancer. These studies performed diagnosis and treatment analysis by measuring the characteristics of overall tumor heterogeneity. For example, the research group of Huang et al. used 132 texture features of CT images to forecast the Disease-Free Survival (DFS) of non–small cell lung cancer (NSCLC) [49], and Goh et al. used fractal dimension features to diagnose and analyze colorectal cancer [75]. However, the heterogeneity features extracted by these methods are basically a measure of the degree of overall tumor heterogeneity (inhomogeneity) based on the grayscale of tumor images, which fails to reflect the basic facts that heterogeneous tumors are composed of tissues with different characteristics. Biomedical analysis of tumors shows that different spatial regions may exhibit changed physiological characteristics [76], leading to specific regions corresponding to different cancer treatment responses, molecular subtypes [77], etc. In order to analyze the heterogeneity of subfunction regions, Diehn et al. selected two regions with high dynamic enhancement rate and low enhancement rate in DCE-MRIs in gliomas. The hypoxia gene expression values of these two tissue regions also showed corresponding high expression values and low expression values; that is, the tumor heterogeneous expression regions are significantly related to imaging characteristics [78]. The first international study explored the correlation between tumor imaging regional features and molecular features. However, the study only detected the heterogeneity between different tumor regions through imaging methods but failed to achieve precise positioning and quantitatively describe the distribution and characteristics of the heterogeneous regions.

In order to accurately locate and describe the imaging heterogeneity of tumor subregions, researchers around the world have made some preliminary attempts to describe the heterogeneity of different tissue characteristics using different imaging modalities [63, 77, 79]. Tumor heterogeneity analysis must first define “content” from the perspective of the image and assign different “attribute” at each voxel to tissue characteristics in the image. For instance, DCE-MRIs measure the status of tumor blood flow and blood vessels; diffusion-weighted images reflect the diffusion and permeability of tumor water molecules; perfusion images measure tumor vascular proliferation, etc. [80] In this way, different tumor tissue characteristics and pathological characteristics can be reflected through a variety of imaging techniques from different perspectives. Taking DCE-MRI as an example, it is reported that DCE-MRIs can be divided into several different representative feature regions according to a certain threshold, and texture features are calculated in these regions to measure the heterogeneity degree of these regions [77, 81, 82]. An increasing number of sophisticated methods cluster similar dynamic enhancement patterns [13, 83, 84] and describe the heterogeneity of vascular characteristics in tumor spaces through DCE-MRIs. But technically, the current stage of tumor heterogeneity analysis is still in its infancy.

As mentioned previously, malignant tumor has become one of the most common diseases harmful to human health, whose precise diagnosis and treatment are studied internationally, but remains unsettled. This paper focused on the precise diagnosis and prognosis prediction of neoadjuvant chemotherapy for cancer disease. Centering the tumor heterogeneity, this paper investigated radiogenomic methods for tumor heterogeneity analysis based on machine learning and explored the relationship between the imaging characteristics and molecular expression characteristics of heterogeneous tumors. A multidimensional MRI radiogenomics data analysis framework was designed based on geometric algebraic representation model to comprehensively explore the rich spatial images, spatial signals, and semantic features in multidimensional multimode MRIs. Besides, a spatial-temporal representation model was designed by focusing on both local and the global feature spaces in different hierarchy, and diversified self-attention mechanisms were implemented. Regarding the heterogeneity of different tumors, this paper proposed an individualized radiogenomic model combining the information about tumor imaging, molecular classification, and tumor clinical treatment for predicting the curative effect of neoadjuvant chemotherapy. It provides scientific guidance for accurate diagnosis, treatment, and prognosis of breast tumor patients, for the purpose of improving the cure rate of the patients with tumor, enhancing the well-being of patients after surgery, and using medical resources effectively and reasonably.

## 6. Conclusions

Tumor heterogeneity is a determinant playing a key role in therapeutic effect and is scarcely known from the perspective of molecular [85]. This paper aims to review the leading research on MRI radiogenomics methods based on the research frontiers in the fields of artificial intelligence and machine learning and focuses on the key core issue of tumor heterogeneity. By analyzing multimodal MR images and molecular information, it is expected to afford methods that can reflect the different functional heterogeneities of tumors. This paper provides a new framework related to temporal-spatial consistent correlation model based on MRI radiogenomics and offers novel intelligent solutions for tumor clinical diagnosis and curative effect prediction in aspects of neoadjuvant chemotherapy, aiming to effectively assist doctors in making correct treatment decisions and improve patients' survival rate and well-being. Two contributions are represented in this paper: (1) an in-depth exploration is conducted for the cross-scale spatial, temporal, and semantic features of multidimensional MR images to be analyzed to reveal the spatial and temporal heterogeneity of tumors with geometric algebra onto radiogenomic methods and achieve correlation analysis from the local functional area to the global semantic space; (2) a novel bidirectional Gated Recurrent Unit (GRU) recurrent neural network (BiGRU-RNN) model is proposed to establish a multidimensional consistent deep learning of tumor heterogeneity with integrating MR imaging parameters and gene expression and predict the curative effect of tumor neoadjuvant chemotherapy.

## Figures and Tables

**Figure 1:** Intertumoral, intratumoral, and time related (temporal) heterogeneity of tumors (from Burrell et al., Nature, 2014 [5]).

**Figure 2:** Introduction of the Two-Stage Intratumoral Partition Framework, that is, stage I: individual level cluster; and stage II: population level cluster, showing the use of matrix originating from intratumor partition diagrams. Quantitative imaging characteristic were obtained from MSI matrix for the sake of the measurement towards the spatial heterogeneity in tumors [51].

**Figure 3:** Framework of the Three-phase Study. Firstly (Phase 1), the nonsupervision deconvolution analysis on gene expression profiles is conducted to recognize prognostic subclone biomarkers. The gene set enrichment analysis is conducted to infer the biological functions of subclones; secondly (Phase 2), radiomic features onto compositions of prognostic subclones are mapped to establish radiogenomic signatures; thirdly (Phase 3), radiogenomic signatures are evaluated on another two independent datasets containing imaging and survival outcomes data [48].

**Figure 4:** Geometric neuron based on McCulloch-Pitts neuron for MRI Imaging Datasets based on General Framework mentioned in References [64, 69] where sp presents a scalar product; {*σ*_*i*_}, *i* = 1, 2,…, *n* orthonormal basis vectors; and gp, geometric product.

**Figure 5:** Framework regarding the association of MRI group and genome based on the analysis of spatial-temporal consistency.

**Figure 6:** BiGRU-RNN network model based on attention. Symbols {*w*_1_,…, *w*_*n*_} are input parameters in relation to MRI radiomics, and the output vectors {*u*_*w*_} and {*u*_*at*_} regard the hidden layer vector {*h*_1_,…, *h*_*n*_} and the radiomics feature vector Vat through the multilayer perceptual network. Similarity matrix *δ* contains the similarities between the genomics vector ug and output attention weight vector *ψ*: namely, the ultimate output of radiogenomics eigenvector is achieved in accordance with the concealed layer vector {*h*_1_,…, *h*_*n*_} and AuGRU weight vector *δ*. Radiogenomic feature fusion is conduced as an AuGRU cell.

**Table 1:** is designed to intuitively classify and introduce the mentioned radiogenomics techniques and approaches in literature for diagnosis, treatment, and prognosis research. The bold text is the categories of radiogenomics techniques for tumor heterogeneity.

**Genome sampling analysis technology for tumor heterogeneity**	Gene expression modules [46].	**Tumor treatment and prognosis research**
Multi-region sampling strategy [6]	Imaging phenotype of the tumor [48, 49]	Predicting NAC efficacy [50, 55–57]
Micro-cutting of tumor tissues [6]	Imaging characteristics of different tumor areas [26]	Survival period [58], distant metastasis [59]
Longitudinal sampling [7–9]	Key tumor genes [27]	Predicate the recurrence-free survival (RFS) [48]
**Radiogenomic approaches for tumor heterogeneity**	Molecular information decomposition [25, 26],	Multiomics approaches [61]
DCE-MRI subcomponent decomposition [26, 27]	Unsupervised convex analysis [6]	**Intratumor heterogeneity**
Unsupervised identification of mixed tissue characteristics [34, 35].	**Radiomics research for tumor heterogeneity**	Multiscale intratumor heterogeneity [48]
Tumor molecular classification [40–42]	Dynamic enhancement rate of fibroglandular mammary glands [33–35]	Perfusion magnetic resonance (MR) imaging via a two-stage intratumor partition framework [51]
